The article "ColoRectalCADx: Expeditious Recognition of Colorectal Cancer with Integrated Convolutional Neural Networks and Visual Explanations Using Mixed Dataset Evidence" was published in 2022. Journal: Comput Math Methods Med.

# ColoRectalCADx: Expeditious Recognition of Colorectal Cancer with Integrated Convolutional Neural Networks and Visual Explanations Using Mixed Dataset Evidence

**DOI:** 10.1155/2022/8723957

**Published:** 2022-11-10

**Authors:** Akella S. Narasimha Raju, Kayalvizhi Jayavel, T. Rajalakshmi

**Affiliations:** ^1^Department of Networking and Communications, School of Computing, SRM Institute of Science and Technology, Kattankulathur, 603203 Chennai, India; ^2^Department of Electronics and Communication Engineering, School of Electrical and Electronics Engineering, SRM Institute of Science and Technology, Kattankulathur, 603203 Chennai, India

## Abstract

Colorectal cancer typically affects the gastrointestinal tract within the human body. Colonoscopy is one of the most accurate methods of detecting cancer. The current system facilitates the identification of cancer by computer-assisted diagnosis (CADx) systems with a limited number of deep learning methods. It does not imply the depiction of mixed datasets for the functioning of the system. The proposed system, called ColoRectalCADx, is supported by deep learning (DL) models suitable for cancer research. The CADx system comprises five stages: convolutional neural networks (CNN), support vector machine (SVM), long short-term memory (LSTM), visual explanation such as gradient-weighted class activation mapping (Grad-CAM), and semantic segmentation phases. Here, the key components of the CADx system are equipped with 9 individual and 12 integrated CNNs, implying that the system consists mainly of investigational experiments with a total of 21 CNNs. In the subsequent phase, the CADx has a combination of CNNs of concatenated transfer learning functions associated with the machine SVM classification. Additional classification is applied to ensure effective transfer of results from CNN to LSTM. The system is mainly made up of a combination of CVC Clinic DB, Kvasir2, and Hyper Kvasir input as a mixed dataset. After CNN and LSTM, in advanced stage, malignancies are detected by using a better polyp recognition technique with Grad-CAM and semantic segmentation using U-Net. CADx results have been stored on Google Cloud for record retention. In these experiments, among all the CNNs, the individual CNN DenseNet-201 (87.1% training and 84.7% testing accuracies) and the integrated CNN ADaDR-22 (84.61% training and 82.17% testing accuracies) were the most efficient for cancer detection with the CNN+LSTM model. ColoRectalCADx accurately identifies cancer through individual CNN DesnseNet-201 and integrated CNN ADaDR-22. In Grad-CAM's visual explanations, CNN DenseNet-201 displays precise visualization of polyps, and CNN U-Net provides precise malignant polyps.

The article "ColoRectalCADx: Expeditious Recognition of Colorectal Cancer with Integrated Convolutional Neural Networks and Visual Explanations Using Mixed Dataset Evidence" was published in 2022. Journal: Comput Math Methods Med.

## 1. Introduction

On a global scale, different people live within their own culture. Their diet differs according to their lifestyle. One way to categorize their eating patterns is to distinguish between vegetarians and nonvegetarians. Despite adopting healthy eating habits and a normal lifestyle, some people are sick. Varieties of diseases are widespread throughout the world, who need doctors specialized in treating these ailments. In India, the patient-physician relationship is 1 : 834 who adopts an allopathic form of treatment. A number of health care professionals in India are practicing Ayurveda, homeopathy, Unani, etc.; 565000 diseases are covered in the treatment of patients [1]. In the US, there are 295 doctors available for 100,000 people [2]. Statistics show that Germany has the highest density of doctors available to patients, where people have a better chance of being treated [3].

Every human being needs health; however, according to their lifestyle and environment, they suffer from a variety of illnesses. Of these diseases, cancer is the most dangerous with a historically high mortality rate. Cancer is a particular type of illness that exhibits abnormal or unhealthy tissue growth (i.e., internal cells) in the internal organs of the body. In humans, it is particularly harmful to blood cells in the organs. The disease develops rapidly over the last few stages, resulting in high mortality rates. Early diagnosis and recognition are critical to improving the survival chances of those living with cancer. There are many types of cancers affecting different organs, such as breast, prostate, basal cell, skin (melanoma), lung, and colon cancer, as well as leukemia and lymphoma [4].

Colon cancer and colorectal cancer (CRC) are the two most dangerous types of cancer in the human gastrointestinal tract. In colorectal cancer, abnormal cells are grown in the large intestine until they get to the rectum. The large intestine is the body's main organ for the digestion of food particles, which is five feet and two inches long. The large intestine can be divided into the ascending, transverse, descending, and sigmoidal colon, and each portion of the colon has a specific function in the process of digestion. Although CRC always starts with little polyps, not all polyps are dangerous. As malignant polyps grow exponentially, they can be converted to cancer in the colon area. This type of cancer is primarily due, for instance, to eating habits, psychological imbalances, and insomnia. The stages of CRC are in situ, local, regional, and distant. First, cancer cells can invade the walls of the colon that can form malignant polyps locally, spread to the wall from the rectum area, and further extend to other parts of the body at an advanced level. The usual symptoms of the disease are bleeding in the rectum and blood in the feces. There are many methods of colon screening to detect CRC or gastrointestinal diseases.

The article "ColoRectalCADx: Expeditious Recognition of Colorectal Cancer with Integrated Convolutional Neural Networks and Visual Explanations Using Mixed Dataset Evidence" was published in 2022. Journal: Comput Math Methods Med.

Among all screening tests, colonoscopy is the reference method for determining the disease [5, 6], which has an accuracy of 95% because in this procedure, the gastroenterologist carries out screening of the entire colon closely. In this procedure, a device called a colonoscope, which is slim and illuminated by a light source equipped with a high-end frontal camera, is used [7]. This device was inserted into the colon through the rectum, and videos and pictures of the whole colon were captured at 5 min intervals and stored on a personal computer (PC). Many of the resulting videos and images are reviewed by a radiologist to determine the area of the colon affected by cancer.

Medical colonoscopy motion images and videos were introduced and used as datasets for new technologies like machine learning (ML) and deep learning (DL) [8]. For early and rapid diagnosis, computing technology may be invoked. In the new technological age, artificial intelligence (AI) plays an important role in automation and robotics. In AI technology, ML and DL are subfields that support new innovations. To be recognized by CRC, the technology supports the combination of biomedical engineering and informatics. Support for deep learning techniques is required to identify cancer for early diagnosis. In DL, we have meticulously conducted investigation experiments with convolutional neural networks (CNNs), which play a major role in this research. CNNs operate within the framework of a computer-assisted diagnosis (CADx), which was developed in various phases to eventually diagnose malignancy. The CADx system, named ColoRectalCADx, is used for CRC diagnosis. Throughout this document, the system is covered under the title “ColoRectalCADx.”

The principal objectives of the study are as follows:

- Design a CRC recognition system through a five-stage process
- The early detection stage is the classification of images through colonoscopy using seven different CNNs. The system presents 12 integrated models of CNN and obtains the most accurate model for cancer classification using three datasets
- End-to-end CNN and fusion models represent transfer learning and SVM classification
- The next phase is the transfer learning of long short-term memory (LSTM). This classification determines the most appropriate cancer recognition model
- There is identification of malignant polyps by Grad-CAM visual explanation
- There is accurate identification of cancer polyps for malignancy recognition: a visualization technique, such as semantic segmentation using the U-Net CNN model, is used at a later stage

The remainder of this paper is organized as follows.  Section 2 provides an overall literature review.  Section 3 describes the materials and the methods.  Section 4 discusses the results, and finally, Section 5 concludes the study.

The article "ColoRectalCADx: Expeditious Recognition of Colorectal Cancer with Integrated Convolutional Neural Networks and Visual Explanations Using Mixed Dataset Evidence" was published in 2022. Journal: Comput Math Methods Med.

## 2. Literature Survey

Duc et al. [9] discussed how polyps in the colorectal regions are recognized effectively and efficiently using new deep learning approaches. The authors proposed an architecture based on deep learning called Colon-Former, which uses an encoder-decoder architecture for recognizing polyps in colonoscopy images as a semantic segmentation concept. The encoder is a lightweight architecture that is used to model global semantic relationships on several scales. The decoder is a hierarchical network that enriches the depiction of image features. For the proposed system, the authors used five reference datasets. This model exploits the benefits of both transformers and CNNs for multiscale functionality representations. However, it operates with only a single architecture and results from five datasets. In addition, the results of the comparisons are considered cutting-edge methods, and we found that it achieved the best results.

Sharma et al. [10] discussed skillful and early detection of precancerous polyps in the area of CRC using ML. The authors proposed a system—an ensemble classifier for the reorganization of malignant polyps in the colorectal area. The proposed system is mainly used for comparison with CNN architecture models, such as ResNet101, GoogleNet, and Xception. This classifier is used as, the first level of detection for informational frame detection, in the next stage, classification to detect polyps in the colon area. In these experiments, the input data were from live Aiche colonoscopy and the Kvasir datasets. Upon comparison of all the results, the proposed ensemble classifier showed an accuracy of 98.3% for the detection of informative images and 97.66% for the recognition of malignant polyps. Nevertheless, the system only compares the three CNN models, whereas there are a number of pretrained models. A real-time dataset and a single publicly accessible dataset were considered for this experiment.

Meng et al. [11] discussed the importance of image segmentation for identifying CRC polyps within the colorectal area using colonoscopy image datasets. Previously, image segmentation was developed using regional dense-pixel classification and polygon methods based on boundaries. The authors introduced a new feature for polyp recognition using a graphical neural network (GNN), which is based on a deep neural network. Using this technique, the polyp region is recognized through an attention-enhancement module (AEM). The AEM supports extraction of the discriminating area and boundary characteristics of the polyps. The GNN functions as the weighted link between the interdomain nodes, and each plot is dependent on the data, which retains the global and local relationships between the nodes. In particular, it addresses the characteristics of the region and boundaries. The GNN outperforms other methods and effectively recognizes malignant polyps in biomedical colonoscopy images. However, the system is very complicated in terms of recognizing the exact polyp area. The comparison system of the numerous leading-edge methods and this specific GNN system is the most suitable model. Only complex objects were used to identify the polyps.

The article "ColoRectalCADx: Expeditious Recognition of Colorectal Cancer with Integrated Convolutional Neural Networks and Visual Explanations Using Mixed Dataset Evidence" was published in 2022. Journal: Comput Math Methods Med.

Kyeong-Beom and Lee [12] suggested a new technique for identifying CRC polyps using different medical colonoscopy datasets. The previously used CNN U-Net architecture has some limitations in the segmentation of medical images. Compared to the previous segmentation, the authors proposed a new encoder-decoder-based architecture called SwinE-Net. It is a new hybrid approach to deep learning for polyp segmentation through a CNN and a Swin transformer. SwinE-Net is an association between the CNN EfficientNet and vision transformer- (ViT-) based Swin transformer. Here, the first convolutional block extracts feature maps to enhance the discriminability of multilevel features of the CNN and ViT. Subsequently, the multifeatured aggregation block creates intermediate outputs of the refined polyp characteristics to be extracted for effective training. Finally, the attentive deconvolutional block rises and works as a decoder to recognize polyp regions in the image datasets. For this SwinE-Net System, experiments were carried out with the five reference datasets, and the polyps of the image datasets were recognized. Nevertheless, the system uses an EfficientNet convolution network. There are other pretrained CNN models that work effectively without using these models, which is too complex to comprehend. The proposed system is compared with previous state-of-the-art technologies, and the best-adapted system is presented as a SwinE-Net model.

Mahanty et al. [13] proposed a new architecture, based on the CNN U-Net called SU-NET, to acknowledge polyps in colonoscopy images using semantic segmentation. It is in the form of a CNN network with an encoder-decoder structure. In this proposed model, most of the top layers transfer pooling inside, and the bottom layers transfer feature maps to incorporate multiscale information for better identification of the contours of the polyp colon. For this experiment, the dataset taken was the CVC Clinic DB. The SU-NET model showed 89.27% accuracy and 0.895 Dice similarity coefficient. However, in this system, we used only one model and conducted experiments with only one dataset. Here, we do not discuss how the performance of complex datasets, such as the number of images at a high pixel level, works.

The article "ColoRectalCADx: Expeditious Recognition of Colorectal Cancer with Integrated Convolutional Neural Networks and Visual Explanations Using Mixed Dataset Evidence" was published in 2022. Journal: Comput Math Methods Med.

Rahim et al. [14] explained that there are numerous techniques for identifying polyps within the concept of image segmentation, but only a small number of techniques provide possible solutions, for obtaining the best adapted method. The authors proposed a deep CNN model that uses a different number of kernels with different window sizes in the hidden layers to extract the specifications. Within this concept, a lightweight model consists of 16 convolutional layers, two fully connected layers, and a SoftMax layer as the output layer is implemented. The activation function MISH is used in the first 15 convolutional layers and then the ReLU activation function. Here, data augmentation for photometric and distortion-level images was used for the input datasets to improve a number of images. The entire experiment achieved possible results for identifying polyps. However, only 196 images from the ETIS-Larib dataset were tested. Here, we do not discuss the number of datasets and the experimentation of the various models. With the augmentation of the dataset from 196 to 2156 images, the solution obtained was 72% nonaugmented image accuracy, which increased to 94.44% accuracy.

Saito et al. [15] presented anatomical images of automatic colonoscopies categorized using deep convolutional neural networks. Colon cancer generally affects parts of the colon, such as the terminal ileum, cecum ascending colon to traverse colon, descending colon to sigmoid colon, rectum, and anus. In the proposed system, a CAD system was developed to determine cancerous cells using CNN classification of various parts of the colon. The CAD system is tested with a different number of colonoscopy images, such as 9995, and obtains the results for the system for every part of the colon. Colonoscopy images were live images taken between January and October 2017. The main CNN model for testing was GoogleNet, which achieved 91.7% accuracy for 507 images. However, only the CNN model is used. There are many other CNN models available, and their performance is not discussed here. There are a few datasets that are not being used.

Zhou and Gao [16] discussed as to how CNN technologies enable intelligent recognition of medical motion images. Earlier, small-scale motion images obtained using traditional recognition techniques were used. Which techniques are time-consuming to compute and require extensive computer statistics? Currently, large-scale intelligent recognition of medical motion images is assisted by CNN algorithms. Here, the features of the dense trajectory are initially learned following the features of depth, and the dense path functions are merged with DL methods. Finally, extreme learning is functional in a CNN, where the descriptions of the bottom layer to the top layer are determined for medical image recognition. However, there are no discussions on obtaining colorectal medical images from colonoscopy screened images and procedure for retrieval and classification of the results according to their image features.

The article "ColoRectalCADx: Expeditious Recognition of Colorectal Cancer with Integrated Convolutional Neural Networks and Visual Explanations Using Mixed Dataset Evidence" was published in 2022. Journal: Comput Math Methods Med.

Attallah and Sharkas [17] proposed a system—Gastro-CADx—to classify several gastrointestinal diseases using DL approaches, consisting of three phases. These four CNNs were used as feature extractors to extract spatial functionality. This study builds upon DL approaches in the next stage of the system. The properties extracted in the first step are applied to the discrete wave transform (DWT) and discrete cosine transform, which are used to extract temporal- and spatial-frequency features. The third step of the system comprises several combinations of characteristics that are merged in a concentrated manner to inspect the effect of the feature combination on the CADx output results and to select the most merged feature set. Two datasets, datasets I and II, respectively, Kvasir and Hyper Kvasir are used to assess the performance of Gastro-CADx. However, this system has been applied to a limited number of datasets. The system is not even under discussion for the semantic segmentation concept of locating and identifying malignant polyps.

Lin et al. [18] introduce the Dual Swin Transform U-Net for Medical Image Segmentation. The automatic segmentation of medical images has come a long way thanks to the development of deep learning. However, most of the available methodologies are based on CNNs. Inspired by the success of Transformer whose self-management mechanism has the powerful ability to model contextual information in the long run, some researchers have put considerable effort into the development of robust transformer-based U-Net variants. The authors present a new deep healthcare image segmentation framework called Dual Swin Transformer U-Net (DS-TransUNet) which could be the first attempt to simultaneously integrate the benefits of Swin Transform hierarchical into the encoder and decoder of the standard U-shaped architecture. Enhance the quality of semantic segmentation of various medical images. Unlike numerous previous Transformer-based solutions, the proposed DS-TransUNet first adopts sub-Swin Transformer based dual-scale encoder networks for extracting representations of course and fine characteristics of different semantic scales. In-depth experiences of four typical medical image segmentation tasks demonstrate the effectiveness of DS-TransUNet and show that our approach greatly exceeds the state-of-the-art methods.

The article "ColoRectalCADx: Expeditious Recognition of Colorectal Cancer with Integrated Convolutional Neural Networks and Visual Explanations Using Mixed Dataset Evidence" was published in 2022. Journal: Comput Math Methods Med.

Jha et al. [19] examine the detection of polyps in real time, location, and segmentation in colonoscopy. For this polyp detection concept, computer-assisted detection and localization and segmentation help to enhance the colonoscopy procedure. The colonoscopy image dataset under consideration here is Kvasir-SEG for the CAD experiment. As a result of the power of deep learning technology, the CAD system is developed here is ColonSegNet. The proposed ColonSegNet achieved a competitive matrix coefficient of 0.8206 and the highest mean speed of 182.38 frames per second for the segmentation task. However, the system is complex and operates on one dataset. How other datasets will be precisely segmented will not be addressed here.

Meena and Roy [20] discuss the detection of bone fractures using deep supervised learning from X-ray imagery. Failed fractures are common prognostic failures in case of accident or emergency. The outcome is complications and delays in treatment and patient care. Nowadays, artificial intelligence (AI) and, more precisely, deep learning (DL) receive considerable attention to help radiologists detect bone fractures. DL can be widely used for diagnostic image analysis. One can conclude that models based on CNN, such as InceptionNet and XceptionNet, are very effective in the case of fracture detection. Diagnostic and prognosis of X-rays by expert radiologists is a lengthy and laborious process that could be computerized using fracture detection techniques. However, the system runs on both CNN models and compares the results with them.

Pal et al. [21] discuss about a fully connected model for automatic segmentation and chest X-ray annotation that is based on UW-Net attention. Automated segmentation and annotation of the medical image play an essential role in scientific research and the medical community. We offered a UW-Net attention, which introduces an intermediate layer acting as a bridge between the encoder and the decoding paths. The intermediate layer is a set of fully connected convolutional layers generated from oversampling, from the final encoder layer connected to the sampled blocks upwards and downwards sampled by unsolicited connections. The intermediary layer is then connected to the decoding channel with a sampling layer. The proposed attention UW-Net is giving a very good performance, achieving an average F1-score of 95.7%, 80.9%, 81.0%, and 77.6% for lung (large), heart (medium), trachea (small), and collarbone (small) object segmentations, respectively. Attention to UW-Net is superior not only in relation to U-Net and its variations but also in relation to other recent automatic and semiautomatic segmentation/annotation models. Consistent predictive accuracy of segmentation masks for all types of segmentation masks (large, medium, and small lesions) makes this model ideal for automatic organ annotation. However, here, the new concept like UW-Net attention is introduced for new segmentation tasks and to compare with advanced methods. It is hard to comprehend new authors.

The article "ColoRectalCADx: Expeditious Recognition of Colorectal Cancer with Integrated Convolutional Neural Networks and Visual Explanations Using Mixed Dataset Evidence" was published in 2022. Journal: Comput Math Methods Med.

Cao et al. [22] discussed implementation of the multicloud framework for the construction of OpenStack—an IoT-based medical platform known as the tristorage error recovery system. Tristorage was conceived as an inherent module in the open stack step and established the native level of management of the multicloud OpenStack platform through a cascading frame. However, large datasets of colonoscopy images are stored in effective cloud technologies, such as AWS clouds, which are not covered here. Therefore, efficient future storage technologies require further investigation.

## 3. Materials and Methods

The key concept in this study is to accelerate the diagnosis of CRC using a CADx, called ColoRectalCADx [23, 24]. ColoRectalCADx consists of five illustration phases for identifying cancer through visual explanations [25]. The phases of ColoRectalCADx are illustrated in Figure 1. The description of the block diagram is as follows.

### 3.1. Colonoscopy Procedure

Colonoscopy is a screening method for diseases of the human gastrointestinal tract, of which colon is the key organ, screened with the aid of a device called a colonoscope. The colonoscope is lightweight and is equipped with a bright frontal camera [26]. The colonoscope is inserted into the colon, which captures photographs and video recording of the four parts of the colon. Colonoscopy was carried out by a gastroenterologist, and the final images and video recordings were reviewed by a radiologist. Finally, the resulting images were considered in our cancer identification research.

### 3.2. Google Cloud

Postcolonoscopy images were categorized based on parts of colon as labelled images called datasets. These images are then stored in the high-end local servers and also in individual account specific Google Cloud [27] and on Google Drive. Extensive research was conducted with the help of Google's colaboratory (Co-Lab) to analyze the results.

The article "ColoRectalCADx: Expeditious Recognition of Colorectal Cancer with Integrated Convolutional Neural Networks and Visual Explanations Using Mixed Dataset Evidence" was published in 2022. Journal: Comput Math Methods Med.

### 3.3. Datasets

The colonoscopy medical motion image datasets used were publicly available image datasets, downloadable from the internet sources: CVC Clinic DB, Kvasir2, and Hyper Kvasir. The datasets were labelled with 2-, 8-, and 23-class labels. In the proposed system, the mixed dataset is the fusion of the CVC Clinic DB [28], Kvasir2 [29], and Hyper Kvasir [30, 31] images in the form of a new mixed dataset containing 24 class labels.

- The CVC Clinic DB dataset included two classes: labelled polyps (818) and non_polyps (822), with a total of 1640 images [28]
- The Kvasir2 dataset includes eight labelled classes: dyed-lifted polyps (1000), dyed-resection margins (1000), esophagitis (1000), normal-cecum (1000), normal-cecum (1000), normal-*z*-line (1000), polyps, and ulcerative colitis (1000), a total of 8000 images [29]
- The Hyper Kvasir dataset includes lower GI tract and upper GI tract, and these two classes of datasets are further classified labelled as 23 classes and called barrettes (42), barrettes-short-segment (53), bbps-0-1 (653), bbps-2-3 (1148), cecum (1009), dyed-lifted-polyps (1003), dyed-resection margins (990), esophagitis-a (404), esophagitis-b-d (260), hemorrhoids (10), ileum (9), impacted stool (132), polyps (1028), pylorus (1000), retroflex-rectum (391), retroflex-stomach (765), ulcerative-colitis-grade-0-1 (35), ulcerative-colitis-grade-1 (201), ulcerative-colitis-grade-1-2 (11), ulcerative-colitis-grade-2 (443), ulcerative-colitis-grade-2-3 (28), ulcerative-colitis-grade-3 (133), and *z*-line (933), a total of 10672 images [30, 31]

The mixed dataset class descriptions are illustrated in Table 1.

The proposed mixed dataset comprised all the 24 classes with a total of 19,621 images. In these, the dataset has 14 classes, out of which the 10 least executed classes are suppressed, with a total of 16,942 images. The data classes removed from the main datasets were barrettes, barrettes-short-segment, esophagitis-b-d, hemorrhoids, ileum, impacted stool, ulcerative-colitis-grade-1, ulcerative-colitis-grade-1-2, ulcerative-colitis-grade-2-3, and ulcerative-colitis-grade-3. Depending on the deletion of certain classes in the dataset, a balanced dataset was obtained. The total mixed dataset images description is explained and illustrated in Figures 2 and 3.

### 3.4. Image Preprocessing

Within this mixed dataset, each labeled class had a different number of frames. The total number of images in the 14 classes came to 16842. Most of these images have different numbers of pixels. These images with different pixel numbers have been converted to a uniform size of 224 × 224 pixels in order to obtain better experimental results. The resized images were subjected to image preprocessing, that is, image augmentation, which was used to increase the number of images. The image augmentation technique included resizing, increasing the zoom range to 0.2, rotational range to 15, and horizontal flip. After image augmentation, the images were divided into training and test sets in the 70 : 30 ratio to get better results. These training and test images were then applied to the CNNs in the next stage of training and testing.

The article "ColoRectalCADx: Expeditious Recognition of Colorectal Cancer with Integrated Convolutional Neural Networks and Visual Explanations Using Mixed Dataset Evidence" was published in 2022. Journal: Comput Math Methods Med.

### 3.5. Image Classification Using CNN

Classification issues in health care and deep learning technology were addressed using CNN. CNNs are extremely helpful for image classification. CNNs are used in the present research with the ColoRectalCADx system, its main role being in identifying CRC. The mixed dataset contains images required to be categorized using the CNN, which takes images as the inputs, subsequent to which, convolution, pooling, activation, dropout, and fully connected to the neural network operations are performed, after which, and classification accuracies are obtained for the images [32, 33]. In the ColoRectalCADx System, investigational experiments were performed with nine individual CNNs: AlexNet, DarkNet-19, ResNet-50V2, DenseNet-201, EfficientNet-B7, VGG-16, VGG-19, NasNetLarge, and InceeptionResNetV2. From these, we have achieved the best CNN precision, which is the most appropriate model for detecting CRC. In addition, with 9 individual models in addition to 12 integrated models, research experiments are carried out to take the best executed model is appropriate to recognize the CRC. See Table 2 for a list of integrated models used in the ColoRectalCADx system.

Each integrated model has been designed by combining different models. In ColoRectalCADx, a total of 21 models were tested, and the best models for the identification of suitable models to be used in the individual and integrated models for CRC were identified. The integrated models in the above table are presented with short names; therefore, in this article, we can follow their suggested names. A CNN was used to classify the input image datasets, as shown in Figure 4. The CNN input is taken as the input image dataset and consists of CVC Clinic DB, Kvasir2, and Hyper Kvasir images. The images were applied to the convolution layer to recover the image features. Additionally, the image features were sent to the max-pooling layer to filter the image values. In the next step, the ReLU activation function was performed, and these values were sent to the fully connected neural network. Finally, the last layer is the SoftMax layer to classify the multiclass classification in order to separate the classes in the input images. The input image may be determined to be a polyp.

The article "ColoRectalCADx: Expeditious Recognition of Colorectal Cancer with Integrated Convolutional Neural Networks and Visual Explanations Using Mixed Dataset Evidence" was published in 2022. Journal: Comput Math Methods Med.

Each individual and integrated model has a clear advantage in the classification of input medical colonoscopy motion images. DL technology is very beneficial for CRC identification. It gives major perceptual vision to successfully and powerfully identifying diseases. Modern studies have found that CNNs can be far deeper, more accurate, and efficient for learning when smaller connections are established between the layers close to the input and those adjacent to the output.  Table 3 provides the total number of parameters for the proposed integrated and individual CNNs and the number of training parameters that work for the CNNs [34].

In the ColoRectalCADx experiment, the system was enabled with the oldest CNN AlexNet model [46, 47]. Furthermore, experiments were carried out on the basis of the oldest AlexNet model at the latest EfficientNet-B7. In these models, investigative experiments were performed with the less-layered CNNs to the highest-number layered CNNs.

All experimental researches on individual and diverse integrated CNNs are applicable to the transfer of learning for further consideration of the mining characteristics. The CNN contains maps that can confine the results of the filter application to an input image dataset. During transfer learning, one of the CNN layers is transferred and replaced by the other. This generally enables the model to work with new aspects added to the model to solve a particular task. The primary objective of transfer learning is to use a model formed from one dataset and transfer knowledge to another [48, 49]. To identify objects using a CNN, the primary convolutional layers of the network are restricted, and only the last layers that make a prediction are formed.

### 3.6. Support Vector Machines

SVM is a core concept in ML that is a supervised learning algorithm [50]. The algorithm is very helpful in classifying, regression, and selecting outliers. It creates a hyperplane which divides the data into various classes. The main objective is to select a hyperplane with the maximum possible limit between the middle vectors in the given dataset [51–53]. SVM recovers the maximum-margin hyperplane and generates hyperplanes for enhanced class isolation. This relates to the binary classification and the multiclass classification [54, 55].

In this study, ColoRectalCADx CNN models are required to convert it into an SVM using the transfer learning concept. The SVM uses a parameter called “kernel_regularizer” that uses the l2 standard and passes the linear function as an activation function in the final output layer. For multiclass classification, it is necessary to use “SoftMax” as activation functionality in SVM. The application of loss is the “square hinge” for multiclass classification. As a result, the last layers of the CNN make modifications, the linear SVM is represented, and the final accuracies of all the CNN from end-to-end and fusion are obtained [56].

The article "ColoRectalCADx: Expeditious Recognition of Colorectal Cancer with Integrated Convolutional Neural Networks and Visual Explanations Using Mixed Dataset Evidence" was published in 2022. Journal: Comput Math Methods Med.

### 3.7. Long Short-Term Memory

LSTM is a type of neural network used in DL, where a recurring neural network functions from time series inputs. LSTM works with time series predictive problems, such as machine translation and voice recognition. Typically, LSTM networks are made up of various blocks, which are called cells. There are two states that go to the following cell: the state of the cell and the hidden state. The memory blocks are responsible for memorizing the manipulations in the memory through the gates. This forget gate is responsible for removing information that is no longer required for the cell status, which was performed using a filtering technique. This allows the performance of the LSTM to be optimized. The input gate is responsible for providing information on the cell state. The output gate is responsible for the absence of the necessary information along the condition of the cell that can be excited at a given time.

In the ColoRectalCADx system, a total of 21 experiments were carried out using different CNNs. These CNN models convert them to LSTM by means of transfer learning. In this CNN, the max pooling layer is replaced by the LSTM model, and the final layer is connected to the SoftMax activation. The final results of all CNN end-to-end and CNN fusion were achieved using LSTM [57].

### 3.8. Visualization Methods

#### 3.8.1. Grad-CAM

After the convolutional neural network is classified, the input images are viewed at the most targeted level to identify the object under consideration. This type of object focusing was referenced using Grad-CAM [58, 59]. This concept uses the object class and gradient information that travel to the final convolutional layer of a CNN. This results in a rough map of the significant areas of the image. Grad-CAM is a rigorous generalization of class activation mapping that enhances the consideration of image classification. This differs from the exact level of pixel gradient visualizations (guided retro-propagation and deconvolutions) during the supervised localization task. When capturing images, finding areas of subtle images without creating pairs of images and texts is often a good practice. The Grad-CAM configuration illustration is shown in Figure 5. The output of the CNN is represented by *Y*^*c*^ class score

(1) $$\begin{array}{c} Y^{c}=\underset{k}{\sum }w_{k}^{c}\frac{1}{Z}\underset{i}{\sum }\underset{j}{\sum }A_{ij}^{k}, \end{array}$$

where *w*_*k*_^*c*^ = 1/*Z*∑_*i*_∑_*j*_*∂Y*^*c*^/*∂A*_*ij*_^*k*^ are the class feature weights, *A*_*ij*_^*k*^ is the feature map, and 1/*Z*∑_*i*_∑_*j*_*A*_*ij*_^*k*^ is the global average pooling.

The article "ColoRectalCADx: Expeditious Recognition of Colorectal Cancer with Integrated Convolutional Neural Networks and Visual Explanations Using Mixed Dataset Evidence" was published in 2022. Journal: Comput Math Methods Med.

Each spatial location (*i*, *j*) of the class-specific saliency map Lc is then computed as the final equation for the discriminatory class saliency map.

(2) $$\begin{array}{c} L_{ij}^{c}=\underset{k}{\sum }w_{k}^{c}.A_{ij}^{k.}. \end{array}$$

In order to perform the polyp focus model in the ColoRectalCADx system, a DL classification model was developed using the dataset. This is a combination of the CVC Clinic DB, Kvasir2, and Hyper Kvasir as a mixed dataset. This mixed medical motion image colonoscopy dataset is as follows: the images are provided as inputs to individual CNN models to get the output image function map. Subsequently, the matrix of the correlative features is sent to the fully connected layer.

To achieve the Grad-CAM results, a heat map of the image was generated from which the Grad-CAM image classification results were generated. These heat maps were superimposed on the resulting CNN colonoscopy images. They were used to classify the images and locate each class in the input images with the corresponding heat map. These should be generated by Grad-CAM images using CNN models. Five CNN algorithms, namely, DenseNet201, EfficientNetB7, VGG16, ResNet50, and VGG19, are used for the Grad-CAM images that are displayed with input medical motion colonoscopy images.

#### 3.8.2. Semantic Segmentation

Each pixel of an object belongs to a special class to which the same label is allocated by the concept of semantic segmentation. This task classifies every pixel in one image with preset classes. Semantic segmentation works primarily on the concept of a mask that involves edge detection. It is the task of the grouped portions of the image which belong to the same class.

The ColoRectalCADx system includes U-Net architecture with data scaling and patch recovery. The combination of Clinc-Seg, KvasirSeg, and Hyper Kvasir as mixed colonoscopy data helps eliminate and recognize malignant cancer polyps. This system allows high polyp detection accuracy and suggests the importance of the U-Net CNN structure with the necessary hyperparameters.

U-Net has been used as the key network architecture for segmentation of medical colonoscopy motion images in ColoRectalCADx [60, 61].  Figure 6 illustrates the structure of the U-Net for semantic segmentation. Its structure can be largely thought of as a network of tail encoders through a network of decoders. The ultimate outcome of this network is the only one that allows semantic segmentation:

- The encoder was the top edge of the framework. Typically, it is a pretrained classification network; it applies convolution blocks trailed by pooling, which is max pooling, and then downsampling to encode the input colonoscopy medical motion images into feature depictions at multiple levels
- The decoder is the second-most extreme of the structure. The objective is to semantically project the discriminatory characteristics (lower resolution) learned by the encoder in the space of pixels, which results in higher image pixels to obtain a solid classification. The decoder involves upsampling and concatenation followed by coherent convolution processes
- Upsampling in CNNs is used for classification and object detection architecture. The perception is that we would intend to reinstate the reduced feature map to the actual original size of the medical colonoscopy motion images, consequently increasing the feature dimensions. Upsampling is also discussed in terms of transposed convolution, upconvolution, or deconvolution

Experimental results for ColoRectalCADx are presented so far. All experiments were carried out with the system hardware specifications, and the software used for this work is shown in the Table 4.

The article "ColoRectalCADx: Expeditious Recognition of Colorectal Cancer with Integrated Convolutional Neural Networks and Visual Explanations Using Mixed Dataset Evidence" was published in 2022. Journal: Comput Math Methods Med.

The essential element of this ColoRectalCADx system is the datasets. Mixed datasets for CVC Clinic DB, Kvasir, and Hyper Kvasir are represented with classes of 14. In each data class, medical colonoscopy motion images are stored and are accessible for CNN training. Details on the datasets are provided in Table 5.

For all the datasets, experimental research with individual CNN and integrated CNN was also conducted with transfer learning by SVM, followed by LSTM. The experiments have been adapted to the hyperparameters. Hyperparameters specific to the whole ColoRectalCADx system are listed in Table 6.

## 4. Results

This study was carried out using a CADx system, called ColoRectalCADx, in five stages. During these five stages, the principal role was played in the investigation experiments of the nine individual CNNs and the twelve integrated CNNs. We compared the overall performance of these 21 CNNs, individually and integrated, and found the best possible model. In these five stages, the results were included in the first stage of the dataset with the individual and integrated CNN experiments. The second stage was a dataset with individual and integrated SVM+CNN experiments. Third stage consisted of the dataset with individual and integrated CNN+LSTM experiments. The fourth stage consisted of a visual explanation using Grad-CAM. Finally, the fifth stage was a visual explanation using semantic segmentation.

The article "ColoRectalCADx: Expeditious Recognition of Colorectal Cancer with Integrated Convolutional Neural Networks and Visual Explanations Using Mixed Dataset Evidence" was published in 2022. Journal: Comput Math Methods Med.

### 4.1. Stage 1: Individual and Integrated CNN Experimentation

In all investigational findings and comparisons, the *mixed dataset* with the individual *CNN DenseNet-201* achieved the best training accuracy of 79.59% and best testing accuracy of 76.31% in agreement with the other CNNs. For all CNNs, the VGG-19 had the lowest train accuracy of 63.38% and the test accuracy of 64.54%.

In all investigational findings and comparisons, the *mixed dataset* with integrated *CNN ADaDR-22* achieved the best training accuracy with *77.42%* testing accuracy is 72.2% in agreement with the other CNNs. For any CNN, the RV-22 displayed the lowest drive accuracy of 34.27% and the test accuracy of 35.69%.

The area under the curve (AUC) is an indicator used to average the performance accuracy of all classes of the datasets and real-positive (TP) and false-positive (FP) values of the dataset classes. These details indicate that less than 50% is the lowest yield in dataset formation. The proposed *mixed dataset* provided the highest AUC accuracy for DenseNet-201, which was 96.76*%* for the individual CNN, and for the integrated CNN ADaDR-22, an AUC accuracy of 95.09% was achieved. The detailed CNN comparison results are presented in Table 7 and Figures 7 and 8.

### 4.2. Stage 2: Individual and Integrated CNN+SVM Experimentation

In all investigational findings and comparisons, the *mixed dataset* with individual *CNN+SVM ResNet-50V2* achieved the best training accuracy of 78.27% and testing accuracy of 78% in agreement with the other CNNs. For any CNN, AlexNet displayed the lowest training accuracy of 30.31% and test accuracy of 30%. The detailed CNN+SVM comparison results are presented in Table 8 and Figures 9 and 10.

In all investigational findings and comparisons, the mixed dataset with integrated CNN+SVM ADaDR-22 achieved the best training accuracy of 82.05% and testing accuracy of 75% in agreement with the other CNNs. For all SVM+CNN, the RV-22 showed the lowest drive accuracy of 63.38% and the test accuracy of 64.54%.

### 4.3. Stage 3: Individual and Integrated CNN+LSTM Experimentation

In all the investigational findings and comparisons, the mixed dataset with individual CNN+LSTM DenseNet-201 achieved the best training accuracy of 87.1% and best testing accuracy of 84.7%, in agreement with the other CNNs. In any CNN+LSTM, the VGG-19 had the lowest drive accuracy of 63.38% and the test accuracy of 64.54%.

The detailed CNN+LSTM comparison results are presented in Table 9 and Figures 11 and 12.

In all the investigational findings and comparisons, the mixed dataset with integrated CNN+LSTM ADaDR-22 achieved the best training accuracy with an 84.61% and best testing accuracy of 82.17%, in agreement with the other CNNs. For any CNN+LSTM, the RV-22 displayed the lowest drive accuracy of 36.76% and test accuracy of 41.43%.

The article "ColoRectalCADx: Expeditious Recognition of Colorectal Cancer with Integrated Convolutional Neural Networks and Visual Explanations Using Mixed Dataset Evidence" was published in 2022. Journal: Comput Math Methods Med.

In the mixed dataset CNN DenseNet-201 model, the classes bbps-0-1, bbps-2-3, cecum, non_polyps, polyps, pylorus, retroflex-rectum, and retroflex-stomach showed ≥90% accuracy with the support of 198, 345, 603, 257, 368, 117, and 230 images, respectively. In the mixed dataset ADaRD-22 CNN-integrated model, some classes showed no (zero) performance with the support of a smaller number of images in the class. Classes bbps-0-1, bbps-2-3, pylorus, retroflex-rectum, and retroflex-stomach have an accuracy of ≥90 percent accuracy with the support of 198, 345, 600, and 230 images, respectively. The performance of the classes is shown in Table 8 and Figure 9. Among all the individual and integrated CNNs, for a total of 21 experiments, the individual CNN DenseNet-201 and integrated CNN ADaDR-22 models showed the best performance. The high-performance individual and integrated CNN models of the individual class performances are shown in detail in Table 10 and Figure 13.

According to the mixed dataset classification results, the best clarifications were obtained with the individual DenseNet-201 CNNs, and for the integrated CNN, ADaDR-22 provided the greatest accuracy. The information is provided by TP, TN, FP, and FN. The corresponding confusion matrices were formed based on the classes described for each dataset. A matrix in the form of a confusion matrix provides a good indication of how well the evaluation model is performing. Every row is a real/true class and every column is a predicted/estimated class. Actual values were compared to those predicted. Thus, for the correct models, many elements are required diagonally. In this case, the confusion matrix has been normalized; so, the value of unit is accepted as the highest value on the diagonal. Our model shows that all classes have diagonal values approaching unity. The confusion matrices corresponding to the highest accuracies are shown in Figure 14.

In order to estimate algorithm recognition performance, they were compared to other medical motion colonoscopy datasets using CNN algorithms. The medical motion image recognition ratio results and ROC curves of the different CNN algorithms obtained the best accuracies with DenseNet-201 for individual CNNs, and for integrated CNNs, ADaDR-22 provided the highest accuracy. The receiver operating characteristic (ROC) curves are presented and illustrated in Figure 15. The recognition rate curves within this multiple-class system classification can be obtained at various levels of accuracy. Based on the accuracies of the CNN, image classes, and ROC graphics, the accuracy class is represented, and the best class of accuracy is discovered and presented in the graphs. These graphs were drawn against the TP and FP rates.

The article "ColoRectalCADx: Expeditious Recognition of Colorectal Cancer with Integrated Convolutional Neural Networks and Visual Explanations Using Mixed Dataset Evidence" was published in 2022. Journal: Comput Math Methods Med.

In this mixed dataset, DenseNet-201 yielded 85–100% accuracy and ADaDR-22 yielded approximately 75–100% accuracy for the 14 classes. In this individual and integrated CNN, both classes are ranked lower to produce a much lower yield.

After the convolutional neural network phase, experimental research on ColoRectalCADx is presented for visual explanations with Grad-CAM and semantic segmentation using the U-Net model. In this study, the Grad-CAM was presented immediately after the CNNs.

### 4.4. Stage 4: Grad-CAM Visualization

To obtain the Grad-CAM results, an image heat map was generated from which the Grad-CAM image classification results were generated. These heat maps are superimposed over the resulting CNN colonoscopy images. They were used to obtain the classification of the images and the localization of each class in the input images with the corresponding heat map, which would have to be generated by Grad-CAM images according to the CNN models. Five CNN algorithms, such as DenseNet201, EfficientNetB7, VGG16, ResNet50, and VGG19, are used for Grad-CAM images and are shown with input medical motion colonoscopy images.

The Grad-CAM results emphasize that they support the area, which implies that these classes concentrate colorectal polyps in the input colonoscopy images. The dark areas are represented in various colors, like red, green, and yellow. These colors displayed on the Grad-CAM output images of the specified classes were displayed due to the prediction of colorectal polyps. This method is useful for discriminating the visual representation of colonoscopy input images to expose the critical area in the image region. The identified zones and features result in significant activation in the upper layers of the colon polyp detection model.

As the guided Grad-CAM rejects bad gradients at every step, it is possible to obtain precise areas of interest for all types of colorectal polyps. Thus, this improved technique helps the doctor to correctly classify the predominant class of polyps and locate several occurrences and different types of polyps on the whole image. CNN classification models were used to detect key polyp detection properties. Therefore, no further training, annotation or segmentation is needed to use visualization methods. The resulting Grad-CAM images using the various CNN models are shown in Figures 16–20, and a comparison of the Grad-CAM images with the various CNN algorithms is given in Table 11. In this DenseNet-201, predicted polyps among other CNNs are precisely identified in mixed datasets.

The article "ColoRectalCADx: Expeditious Recognition of Colorectal Cancer with Integrated Convolutional Neural Networks and Visual Explanations Using Mixed Dataset Evidence" was published in 2022. Journal: Comput Math Methods Med.

Following the main visual explanation with Grad-CAM, the major discovery of malignant CRC polyps was found with semantic segmentation using U-Net.

### 4.5. Stage 5: Semantic Segmentation Using U-Net Visualization

This ColoRectalCADx system in the final stage was used to identify and recognize real polyps that are malignant with the combination of three types of datasets, such as CVC Clinic-Seg, KvasirSeg, and Hyper Kvasir, as a mixed dataset segmentation. The mixed dataset provided inputs for the ColoRectalCADx system, which was integrated into the U-Net CNN structure. U-Net runs as a CNN on an encoder-decoder network. The learning rate was set to 0.001, batch size of the images was 64, and epochs were set to 40. The resulting training and testing losses are listed in Table 12.

For each of the three datasets, the original images with the corresponding mask of the images and malignant polyps are recognized accurately with training losses. The predicted final polyp obtained with the ColoRectalCADx system is depicted in the Figure 21.

The system accurately and effectively identified malignant polyps in all input datasets containing various polyps. The anticipated polyp was the true recognition of polyps. The corresponding loss and epoch graphs are shown in Figure 22.

## 5. Discussion

The ColoRectalCADx system essentially works with the 9 individual CNN models and 12 integrated CNN models. With a total of 21 experiments, the individual CNN DenseNet-201 and the integrated CNN ADaDR-22 provide accurate optimization for detecting colorectal cancer. Primary inputs are mixed datasets, whereas these datasets are integrated with individual datasets.  Table 13 illustrates how individual datasets are executed and the CNN model which shows optimization performance.

This ColoRectalCADx system works with mixed datasets inputs, which is a combination of CVC Clinic DB, Kvasir2, and Hyper Kvasir. This system now provides the highest individual CNN performance achieved by DenseNet-201 with 87.1% and 84.7% training and test accuracy, respectively. The integrated CNN ADaDR-22 reached training and test accuracy of 84.61% and 82.17%, respectively. The system ends with the CNN+LSTM combination, yielding an exact output. Prior to experimentation with mixed datasets, the system also operated with individual dataset inputs and obtained the results for each dataset autonomously. Using the CVC Clinic DB dataset for the individual CNN, DenseNet-201 achieved the highest training and test accuracy of 95.37% and 99%, respectively. The system also works with the integrated CNN DarD-22, with the highest training and test accuracy of 93.86% and 96%, respectively. Using the Kvasir dataset for the Individual CNN, DenseNet-201 achieved the highest training and test accuracy of 80.53% and 88%, respectively. The system also operates with the integrated DarD-22 CNN, with the highest drive and test accuracy of 77.01% and 82%, respectively. Using the Hyper Kvasir dataset for the individual CNN, DenseNet-201 obtained the highest training and test accuracy of 78.17% and 84%, respectively. The system also operates with the built-in DarD-22 CNN, with the highest training and test accuracy of 62.38% and 66%, respectively. For these three datasets, the system results were combined with those of CNN, DWT, and SVM. All information on mixed and individual datasets and the best results achieved are presented in Table 13 and Figure 23.

The article "ColoRectalCADx: Expeditious Recognition of Colorectal Cancer with Integrated Convolutional Neural Networks and Visual Explanations Using Mixed Dataset Evidence" was published in 2022. Journal: Comput Math Methods Med.

The results from the entire ColoRectalCADx system were compared with the three-step GastroCADx system proposed in 2021. Results for all three datasets are presented in Table 14. In GastroCADx, the system was compared to four end-to-end CNN models, but in ColoRectalCADx, it was compared to seven end-to-end CNN models. GastroCADx proved that ResNet-50 was the most appropriate model, and DenseNet-201 was the best model for the ColoRectalCADx system. In comparison, the two systems were nearly identical, but the behavior of the tasks was different. Different system models, such as ensemble classifier, DP-CNN, and MP-FSSD, are discussed starting in 2021 and 2022 and compared with ColoRectalCADx. The previous ColoRectalCADx system was 98%, 88%, and 84% accurate with 3 datasets, respectively. The proposed new system with a mixed dataset was 84.7% accurate.

As a visual explanation, the Grad-CAM operates rather than the max pooling layer of the CNN. In this case, CNN such as DenseNet201, EfficientNetB7, VGG16, ResNet50, and VGG19 is used for Grad-CAM images and is displayed with the input medical motion colonoscopy images. Each CNN provides Grad-CAM output images for the input mixed colonoscopy image dataset. Consequently, the best visualization and localization of polyps are obtained from the CNN DenseNet-201. In each image, it precisely demonstrates malicious polyps are perfectly recognized.

In semantic segmentation, the system operates on the CNN U-Net which is an encoder-decoder network. The input images are applied to the encoder section while the output images are derived from the decoder part. Within the whole image dataset where the polyp images are present, they can be predicted as polyps as image segmentation. Therefore, the ColoRectalCADx system will accurately recognize colorectal cancer using the CNN classification method and spot visual explanation methods with mixed datasets. The Kvasir-SEG dataset assessment criteria are shown in Table 15 and Figure 24.

The article "ColoRectalCADx: Expeditious Recognition of Colorectal Cancer with Integrated Convolutional Neural Networks and Visual Explanations Using Mixed Dataset Evidence" was published in 2022. Journal: Comput Math Methods Med.

## 6. Conclusion

CRC is the third largest cancer type in the world. Colonoscopy screening is an important part of detecting cancer. The datasets have been retrieved from the colonoscopy images. The public-access colonoscopy datasets selected for this research were the CVC Clinic DB, Kvasir, and Hyper Kvasir, which are 2.8.23 classes. Each class contains a separate number of clinical motion colonoscopy images. These three datasets are combined to create a new dataset called mixed datasets, which has a total of 24 classes including 19,621 images, and after modification with balanced classes, it has 14 classes including 16,942 images. The CADx system, referred to as ColoRectalCADx, was designed to recognize cancer. This CADx system is composed of five stages, namely, CNNs, SVM, LSTM, and visual methods, like Grad-CAM and semantic segmentation. ColoRectalCADx inputs were captured from the mixed medical motion image datasets. Once the datasets are stored in Google Cloud, the image preprocessing steps are completed. Subsequently, the main and central parts of cancer recognition began with the CNN process, which was completed with 9 individual CNNs and 12 integrated CNNs for the classification process. The nine individual CNNs were the well-known pretrained models. Moreover, they have been combined into integrated models. With all 21 CNNs, experiments were conducted to determine the most precise and suitable model for CRC recognition. In these experimental investigations, of all CNNs, the individual CNN DenseNet-201 (87.1% training and 84.7% testing accuracies, respectively) and the integrated CNN ADADR-22 (84.61% training and 82.17% testing accuracies, respectively) were the most efficient for cancer detection with the CNN+LSTM model. After CNN, SVM, and LSTM, visualization methods, such as Grad-CAM visualization of the focused class of the input mixed dataset images, are presented for the identification of malignant polyps in cancer images. DenseNet-201 provided the most accurate images for cancer detection. In the final stage of the system, medical colonoscopy datasets are in the process of locating and identifying malignant polyps. For all images of the three datasets, semantic segmentation using the U-Net CNN structure recognizes malignant polyps. For that loss score, the mixed dataset was 0.4223. Semantic segmentation identified the polyps of origin with the predicted malignant polyps.

In a future work, the same experiments will be carried out and enhanced for all clinical colonoscopy motion video datasets. Video datasets represent the number of frames to be taken into account. In this case, the images are augmented in relation to the image datasets so that those video datasets reach a much higher level.

The article "ColoRectalCADx: Expeditious Recognition of Colorectal Cancer with Integrated Convolutional Neural Networks and Visual Explanations Using Mixed Dataset Evidence" was published in 2022. Journal: Comput Math Methods Med.

## Figures and Tables

**Figure 1:** The block diagram of the ColoRectalCADx system.

**Figure 2:** Mixed dataset representation.

**Figure 3:** Sample mixed dataset.

**Figure 4:** CNN architecture.

**Figure 5:** Steps for Grad-CAM localization of images.

**Figure 6:** Semantic segmentation using U-Net.

**Figure 7:** Individual CNN comparison of accuracy metrics are illustrated.

**Figure 8:** Integrated CNN comparison of accuracy metrics is illustrated.

**Figure 9:** Individual CNN+SVM comparison of accuracy metrics is illustrated.

**Figure 10:** Integrated CNN comparison of accuracy metrics is illustrated.

**Figure 11:** Individual CNN+LSTM comparison of accuracy metrics is illustrated.

**Figure 12:** Integrated CNN+LSTM comparison of accuracy metrics is illustrated.

**Figure 13:** High-performance CNN class accuracies.

**Figure 14:** The confusion matrices of mixed datasets.

**Figure 15:** The ROC curves of mixed datasets.

**Figure 16:** Grad-CAM results of the CNN model DenseNet-201.

**Figure 17:** Grad-CAM results of the CNN model EfficientNet-B7.

**Figure 18:** Grad-CAM results of the CNN model VGG-16.

**Figure 19:** Grad-CAM results of the CNN model VGG-19.

**Figure 20:** Grad-CAM results of the CNN model ResNet-50 V2.

**Figure 21:** Semantic segmentation for predicted polyps of mixed dataset.

**Figure 22:** Loss graph of semantic segmentation for mixed dataset.

**Figure 23:** All datasets perform best.

**Figure 24:** Qualitative results comparison on the Kvasir-SEG dataset. From the left: (1) image, (2) ground truth, (3) U-Net, (4) ResU-Net, (5) ResU-Net-mod, (6) ResU-Net++, and (7) U-Net (ours). From the experimental results, we can say that U-Net produces better segmentation masks than other competitors.

**Table 1:** Class labels of the mixed dataset.

Classes	Original mixed dataset	Images	Modified classes	Modified mixed dataset	Images
0	Barretts	42	0	bbps-0-1	653
1	Barretts-short-segment	53	1	bbps-2-3	1148
2	bbps-0-1	653	2	Cecum	2009
3	bbps-2-3	1148	3	Dyed-lifted-polyps	2003
4	Cecum	2009	4	Dyed-resection-margins	1990
5	Dyed-lifted-polyps	2003	5	Esophagitis-a	1404
6	Dyed-resection-margins	1990	6	Non_polyps	818
7	Esophagitis-a	1404	7	Polyps	2150
8	Esophagitis-b-d	260	8	Pylorus	2000
9	Hemorrhoids	10	9	Retroflex-rectum	391
10	Ileum	9	10	Retroflex-stomach	765
11	Impacted-stool	132	11	Ulcerative-colitis-grade-0-1	1035
12	Non_polyps	818	12	Ulcerative-colitis-grade-2	443
13	Polyps	2150	13	*z*-line	1933
14	Pylorus	2000			
15	Retroflex-rectum	391			
16	Retroflex-stomach	765			
17	Ulcerative-colitis-grade-0-1	1035			
18	Ulcerative-colitis-grade-1	201			
19	Ulcerative-colitis-grade-1-2	11			
20	Ulcerative-colitis-grade-2	443			
21	Ulcerative-colitis-grade-2-3	28			
22	Ulcerative-colitis-grade-3	133			
23	*z*-line	1933			
		19621			16942

The article "ColoRectalCADx: Expeditious Recognition of Colorectal Cancer with Integrated Convolutional Neural Networks and Visual Explanations Using Mixed Dataset Evidence" was published in 2022. Journal: Comput Math Methods Med.

**Table 2:** Integrated models and their suggested names.

S. no.	Integrated models	Suggested name
1	AlexNet+DarkNet-19+ResNet-50v2+DenseNet-201+EfficientNet-B7+VGG-16+VGG-19+InceptionResNetV2	ADaRDEV^2^I-22
2	AlexNet+DarkNet-19+ResNet-50v2+DenseNet-201+EfficientNet-B7+VGG-16+VGG-19	ADaRDEV^2^-22
3	ResNet-50v2+DensNet-201+EfficientNet-B7+VGG-16+VGG19	RDEV^2^-22
4	AlexNet+DarkNet-19+DenseNet-201+ResNet-50V2	ADaDR-22
5	AlexNet+DarkNet+ResNet-50V2	ADaR-22
6	DarkNet-19+ResNet-50V2+DenseNet-201	DaRD-22
7	DensNet-201+EfficientNet-B7+VGG-16	DEV-22
8	AlexNet+DarkNet-19	ADa-22
9	ResNet-50V2+DensNet-201	RD-22
10	ResNet-50V2+VGG19	RV-22
11	AlexNet+DenseNet-201	AD-22
12	DarkNet-19+ResNet-50V2	DaR-22

**Table 3:** Number of CNN parameters of CNNs.

CNN architecture models	Introduced year	Total params	Trainable params	Nontrainable params	Layers
AlexNet [35, 36]	2012	2,81,02,775	2,80,81,639	21,136	23
DarkNet-19 [37]	2017	1,60,45,847	1,60,32,983	12,864	19
ResNet-50v2 [38]	2016	2,59,33,975	23,69,175	2,35,64,800	50
DenseNet-201 [39] [40]	2018	1,94,29,463	11,07,479	1,83,21,984	201
EfficientNet-B7 [41]	2019	6,55,73,799	14,76,119	6,40,97,680	813
VGG-16 [42]	2014	1,53,14,391	5,99,703	1,47,14,688	16
VGG-19 [43]	2014	2,06,24,087	5,99,703	2,00,24,384	13
NasNetLarge [44]	2018	87,256,682	2,339,864	84,916,818	414
InceptionResNetV2 [45]	2016	55,398,648	1,061,912	54,336,736	164
Proposed integrated models					
ADaRDEV^2^I-22	2022	246,429,456	71,359,568	175,069,888	
ADaRDEV^2^-22		19,10,28,063	7,02,94,911	12,07,33,152	
RDEV^2^-22		14,68,78,383	2,61,79,231	12,06,99,152	
ADaDR-22		8,94,87,664	4,75,66,880	4,19,20,784	
ADaR-22		2,59,33,000	23,68,200	2,35,64,800	
DaRD-22		6,13,99,840	1,95,00,192	4,18,99,648	
DEV-22		100,319,600	3,185,248	97,134,352	
ADa-22		4,41,26,048	4,40,92,048	34,000	
RV-22		46,559,368	22,994,568	23,564,800	
RD-22		4,53,61,624	34,74,840	4,18,86,784	
AD-22		4,75,16,384	2,91,73,264	1,83,43,120	
DaR-22		4,19,67,694	1,83,90,030	2,35,77,664	

**Table 4:** System specifications.

System	Precision tower T5810
Company	Dell
Processor	Intel® Xeon® CPU core i7 E5-2630
Speed	2.20 GHZ
RAM	32 GB
GPU	GPU NVIDIA Xp.
Software Environment	Google ColabPro+ with Python 3.7.12
Software Python packages	Keras and TensorFlow 2.7.0

**Table 5:** Train and test split of three datasets.

Datasets	Training set	Test sets	Total images
Mixed datasets	12885	4,057	16,942

The article "ColoRectalCADx: Expeditious Recognition of Colorectal Cancer with Integrated Convolutional Neural Networks and Visual Explanations Using Mixed Dataset Evidence" was published in 2022. Journal: Comput Math Methods Med.

**Table 6:** Hyperparameters for the ColoRectalCADx system.

Dataset	Epochs	Batch sizes	Learning rate	Optimizer	Momentum	Dropout
Mixed datasets	30	16	0.0001	Adam	0.9	0.5

**Table 7:** Comparison of accuracies and AUC for various CNN architectures.

Individual CNN	CNN training accuracy in %	CNN testing accuracy in %	AUC in %
AlexNet	80.86	72.3	96.62
DarkNet-19	77.55	61.95	95.62
ResNet-50v2	73.41	75.78	96.37
DenseNet-201	79.59	76.31	96.76
EfficientNet-B7	62.48	70.67	95.7
VGG-16	67.51	66.78	95.64
VGG-19	63.38	64.54	94.59
NasNetLarge	79.67	71.14	96.46
InceptionResNetV2	79.71	74.44	96.57

Integrated CNN	CNN training accuracy in %	CNN testing accuracy in %	AUC in %
ADaRDEV^2^I-22	76.32	72.2	96.16
ADaRDEV^2^-22	72.11	69.85	95.46
RDEV^2^-22	73.57	70.75	94.89
ADaDR-22	77.42	72.2	95.09
ADaR-22	67.55	63.6	94.4
DaRD-22	72.59	72.13	95.28
DEV-22	61.71	61.13	94.66
ADa-22	59	54.61	93.04
RD-22	68.26	67.53	94.46
RV-22	34.27	35.69	84.8
AD-22	71.96	64.13	94.44
DaR-22	70.15	66.59	91.96

**Table 8:** Comparison of accuracies of CNN+SVM architectures.

Individual CNN	CNN+SVM training accuracy	CNN+SVM testing accuracy
AlexNet	44.33	45
DarkNet-19	77.69	72
ResNet-50v2	78.27	78
DenseNet-201	74.29	73
EfficientNet-B7	48.15	60
VGG-16	70.07	65
VGG-19	63.96	65
NasNetLarge	73.47	68
InceptionResNetV2	78.1	69

Integrated CNN	CNN+SVM training accuracy	CNN+SVM testing accuracy
ADaRDEV^2^I-22	67.92	66
ADaRDEV^2^-22	69.45	57
RDEV^2^-22	69.51	69
ADaDR-22	82.04	75
ADaR-22	63.31	64
DaRD-22	68.68	66
DEV-22	61.82	67
ADa-22	58.21	51
RD-22	61.81	64
RV-22	30.31	30
AD-22	66.47	65
DaR-22	60.53	59

**Table 9:** Comparison of accuracies of CNN+LSTM architectures.

Individual CNN	CNN+LSTM training accuracy in %	CNN+LSTM testing accuracy in %
AlexNet	86.81	77.56
DarkNet-19	83.46	68.51
ResNet-50v2	79.57	83.21
DenseNet-201	87.1	84.7
EfficientNet-B7	67.53	77.56
VGG-16	72.7	71.76
VGG-19	69.46	70.16
NasNetLarge	83.57	78.1
InceptionResNetV2	84.52	80.36

Integrated CNN	CNN+LSTM training accuracy	CNN+LSTM testing accuracy
ADaRDEV^2^I-22	81.43	81.9
ADaRDEV^2^-22	78.56	78.56
RDEV^2^-22	79.54	77.01
ADaDR-22	84.61	82.17
ADaR-22	73.23	70.57
DaRD-22	76.84	79.56
DEV-22	64.82	67.98
ADa-22	62.32	60.19
RD-22	73.1	64.6
RV-22	36.76	41.43
AD-22	78.15	67.83
DaR-22	74.26	72.94

**Table 10:** Comparison of precision and support of mixed dataset classes.

Classes		High-performance CNN models		
		DenseNet-201	ADaDR-22	Support
		Precision	Precision	
0	bbps-0-1	0.97	0.92	198
1	bbps-2-3	0.99	0.96	345
2	Cecum	0.9	0.72	603
3	Dyed-lifted-polyps	0.55	0.58	601
4	Dyed-resection-margins	0.77	0.79	597
5	Esophagitis-a	0.43	0	421
6	Non_polyps	0.97	0.84	257
7	Polyps	0.96	0.68	368
8	Pylorus	0.89	0.9	600
9	Retroflex-rectum	0.94	1	117
10	Retroflex-stomach	0.98	0.97	230
11	Ulcerative-colitis-grade-0-1	0.34	0	311
12	Ulcerative-colitis-grade-2	0.37	0.3	133
13	*z*-line	0.63	0.58	580

The article "ColoRectalCADx: Expeditious Recognition of Colorectal Cancer with Integrated Convolutional Neural Networks and Visual Explanations Using Mixed Dataset Evidence" was published in 2022. Journal: Comput Math Methods Med.

**Table 11:** Comparison of Grad-CAM images with CNN algorithms.

Dataset	Images in dataset	Classes in dataset	CNN architecture	Grad-CAM output obtained	Grad-CAM Polyp Prediction
Mixed dataset	19,621	24	VGG16	Yes	High
			VGG19	Yes	Moderate
			ResNet50	Yes	Moderate to high
			DenseNet201	Yes	Very high
			EfficientNetB7	Yes	Low

**Table 12:** Parameters of U-Net for semantic segmentation.

Dataset	Epochs	Learning rate	Batch size	Train loss	Test loss	Total time taken for model
Mixed dataset	40	0.001	64	0.3176	0.4223	2201.05 s

**Table 13:** Comparison of best results of individual and mixed datasets.

Dataset	Model type	Model	Training accuracy in %	Testing accuracy in %
CVC Clinic DB	Individual CNN	CNN+DWT+SVM (DenseNet-201)	95.37	99
	Integrated CNN	CNN+DWT+SVM (DaRD-22)	93.86	96

Kvasir2	Individual CNN	CNN+DWT+SVM (DenseNet-201)	80.53	88
	Integrated CNN	CNN+DWT+SVM (DaRD-22)	77.01	82

Hyper Kvasir	Individual CNN	CNN+DWT+SVM (DenseNet-201)	78.17	84
	Integrated CNN	CNN+DWT+SVM (RDEV2-22)	62.38	66

Mixed dataset (CVC Clinic DB+Kvasir2+Hyper Kvasir)	Individual CNN	CNN+LSTM (DenseNet-201)	87.1	84.7
	Integrated CNN	CNN+LSTM (ADaDR-22)	84.61	82.17

**Table 14:** Comparison of the results of previous state-of-the-art methods from 2021 to 2022.

Dataset	Author	Method	Accuracy in %
CVC Clinic DB	Attallah and Sharkas [17]	GastroCADx	—
	Liew et al. [62]	Ensemble classifier (ResNet50+AdaBoost)	97.91
	Sharma et al. [10]	Ensemble classifier	98.3
	Nisha et al. [63]	DP-CNN	99.6
	Souaidi and El Ansari [64]	MP-FSSD	91.56
	Ours	ColoRectalCADx(previous)	99

Kvasir2	Attallah and Sharkas [17]	GastroCADx	97.3
	Sharma et al. [10]	Ensemble classifier	97
	Ours	ColoRectalCADx (previous)	88

Hyper Kvasir	Attallah and Sharkas [17]	GastroCADx	99.7
	Ours	ColoRectalCADx (previous)	84

Mixed dataset	Ours	ColoRectalCADx (proposed)	84.7

**Table 15:** Comparison of the results of previous state-of-the-art methods of Kvasir-SEG dataset.

Method	Dice coefficient
ResU-Net++ [65]	0.8133
ResU-Net-mod	0.7909
ResU-Net	0.5144
U-Net	0.7147
U-Net (ours)	0.8129

## Data Availability

Data are available in the following links: “https://www.kaggle.com/balraj98/cvcclinicdb” 2015 [Online] [Accessed 25 May 2021], “https://datasets.simula.no/kvasir/” 2016 [Online] [Accessed 3 July 2021], and “https://datasets.simula.no/hyper-kvasir/” 2020 [Online] [Accessed 3 July 2021].
